# Proliferation and survival of human amniotic epithelial cells during their hepatic differentiation

**DOI:** 10.1371/journal.pone.0191489

**Published:** 2018-01-18

**Authors:** Julieta L. Maymó, Rodrigo Riedel, Antonio Pérez-Pérez, Marta Magatti, Bernardo Maskin, José Luis Dueñas, Ornella Parolini, Víctor Sánchez-Margalet, Cecilia L. Varone

**Affiliations:** 1 Universidad de Buenos Aires, CONICET, Instituto de Química Biológica de la Facultad de Ciencias Exactas y Naturales (IQUIBICEN), Ciudad Universitaria Pabellón 2, 4° piso, (1428), Buenos Aires, Argentina; 2 Universidad de Buenos Aires, Facultad de Ciencias Exactas y Naturales, Departamento de Química Biológica, Ciudad Universitaria Pabellón 2, 4° piso, (1428), Buenos Aires, Argentina; 3 Departamento de Bioquímica Médica y Biología Molecular, Hospital Universitario Virgen Macarena, Facultad de Medicina, Universidad de Sevilla, Avenida Sánchez Pizjuán 4 (41009), Sevilla, España; 4 Centro di Ricerca E. Menni- Fondazione Poliambulanza- Istituto Ospedaliero, Brescia, Italia; 5 Hospital Nacional Profesor Alejandro Posadas, Buenos Aires, Argentina; 6 Servicio de Ginecología y Obstetricia, Hospital Universitario Virgen Macarena, Sevilla, España; Shanghai Jiao Tong University, CHINA

## Abstract

Stem cells derived from placental tissues are an attractive source of cells for regenerative medicine. Amniotic epithelial cells isolated from human amnion (hAECs) have desirable and competitive characteristics that make them stand out between other stem cells. They have the ability to differentiate toward all three germ layers, they are not tumorigenic and they have immunosuppressive properties. Although liver transplantation is the best way to treat acute and chronic hepatic failure patients, there are several obstacles. Recently, stem cells have been spotlighted as alternative source of hepatocytes because of their potential for hepatogenic differentiation. In this work, we aimed to study the proliferation and survival of the hAECs during their hepatic differentiation. We have also analyzed the changes in pluripotency and hepatic markers. We differentiated amniotic cells applying a specific hepatic differentiation (HD) protocol. We determined by *q*RT-PCR that hAECs express significant levels of SOX-2, OCT-4 and NANOG during at least 15 days in culture and these pluripotent markers diminish during HD. SSEA-4 expression was reduced during HD, measured by immunofluorescence. Morphological characteristics became more similar to hepatic ones in differentiated cells and representative hepatic markers significantly augmented their expression, measured by *q*RT-PCR and Western blot. Cells achieved a differentiation efficiency of 75%. We observed that HD induced proliferation and promoted survival of hAECs, during 30 days in culture, evaluated by ^3^H-thymidine incorporation and MTT assay. HD also promoted changes in hAECs cell cycle. Cyclin D1 expression increased, while p21 and p53 levels were reduced. Immunofluorescence analysis showed that Ki-67 expression was upregulated during HD. Finally, ERK 1/2 phosphorylation, which is intimately linked to proliferation and cell survival, augmented during all HD process and the inhibition of this signaling pathway affected not only proliferation but also differentiation. Our results suggest that HD promotes proliferation and survival of hAECs, providing important evidence about the mechanisms governing their hepatic differentiation. We bring new knowledge concerning some of the optimal transplantation conditions for these hepatic like cells.

## Introduction

One of the biggest challenges of regenerative medicine is to find a safe and effective source of stem cells that can be used for treatment of different diseases. Although embryonic and adult stem cells represent a promise for the cure or correction of structural, congenital or acquired diseases, there are limitations in their use in clinical practice. They have ethical and legal obstacles, they are difficult to obtain and tumorigenicity has been associated. In recent years much attention has been given to the diverse cell types that can be isolated from the placenta, which is now recognized as a rich and plentiful source of pluripotent and multipotent stem cells. Gestational tissue offers considerable advantages over other sources of stem cells: the unlimited potential supply of, the easy access to such tissues, minimal ethical and legal barriers associated with their use, they can be obtained without the need of invasive procedure and more importantly, they are not tumorigenic [1, 2]. Furthermore, placental stem cells have unique and valuable immunomodulatory properties [3].

Fetal membranes are composed by the amnion, the chorion and the decidua capsularis [4]. The amniotic membrane is formed by an epithelial layer, in contact with the amniotic fluid, resting on connective tissue and a spongy collagenous layer containing mesenchymal cells [1]. Two types of stem cells can be isolated from the human amniotic membrane: the amnion mesenchymal stromal cells (hAMSCs), sparsely distributed in the stroma, and the epithelial amniotic cells (hAECs). HAECs line the inner of two fetal derived membranes attached to the placenta. They arise from the pluripotent epiblast, which give rise to all three germ layers of the embryo [5]. Since the epiblast is formed in the early stage of embryogenesis, immature undifferentiated cells could be found. Thus, isolated hAECs express markers normally present on embryonic cells or germ cells [6, 7]. Notably, primary hAECs have several features that make them most attractive for cellular therapies. Likewise the known advantages of the placental tissues for regenerative medicine, hAECs have other important properties that have contributed to their promising potential in that field, mainly their ability to differentiate into all three germ layers, their low immunogenicity and the anti-inflammatory properties [8–12]. Amniotic stem cells not only lack telomerase expression but also they are non tumorigenic when transplanted [7]. They express stem cell surface markers, such as stage specific embryonic antigen-4 (SSEA-4) and SSEA-3 and tumor rejection antigen 1–60 (TRA1-60) and TRA1-81, which are known to be expressed in human embryonic stem (hES) cells [13]. Concerning pluripotency, specific related molecular markers like NANOG, the octamer-4 (OCT-4), Lefty-A, sex determining region Y-box 2 (SOX-2), teratocarcinoma-derived growth factor 1 (TDGF-1), were found expressed in hAECs [14]

Amniotic epithelial cells have been reported to differentiate into a broad spectrum of cell types. They are capable to origin insulin secreting pancreatic β-islet like-cells [15], functional neurons and glia [16–18] and surfactant producing alveolar epithelial cells [19, 20]. Several laboratories have also reported hepatic [20–23], cardiac [24], osteogenic [9], chondrogenic [25] and adipogenic [9] differentiation of hAECs. Among others attractive features for the clinic, the amniotic membrane promotes re-epithelization, inhibits angiogenesis, decreases inflammation and is used in ocular surface reconstruction and in wounds healing [26].

Liver diseases affect millions of people all over the world. The only currently available curative treatment for end stage liver disease arising from chronic exposure to viruses, excessive alcohol use, metabolic diseases and acute liver failure is orthotropic liver transplantation [27]. However, due to the severe shortage of suitable donor organs and the need for life-long immune suppression following transplantation, alternative therapies are being actively investigated. In the last years, the rise of knowledge concerning not only the biology of the stem cells but also the processes for liver repair has unraveled new ways for the use of stem cells in liver regenerative medicine. Despite the existence of several types of stem cells that can differentiate into hepatic like cells [28], hAECs seem to be ideal candidates.

Placental stem cells not only expressed some features of human liver cells, but also demonstrated several functions of typical hepatocytes [29, 30]. Under specific culture conditions hAECs could adopt hepatic characteristics. Moreover, some studies have reported that freshly isolated hAECs show primitive hepatic differentiation in culture [23, 31]. Previous studies suggested that human amnion membrane or isolated epithelial cells could be safely transplanted into animals or patients and they could be useful in the treatment of liver diseases [32–35].

Encouraged by the known advantages, diverse studies have dedicated their efforts to find new protocols or to optimize the developed ones to have mature hepatocytes from undifferentiated hAECs [21, 23, 31, 36–38]. What it would be preferred is to find the right time during the culture and differentiation of hAECs, so they could be as efficient as possible when being used in the clinic. In this context, there is a lack of studies about the molecular and cellular processes that occur during the hepatic differentiation of amniotic stem cells. Furthermore, a few works have investigated about the biology of the hAECs themselves. Indeed, despite the advantages related to the use of hAECs as stem cells, several limitations remain unsolved, as large numbers of cells are required for its application in transplantation and tissue engineering [7]. The yield of cells obtained per amnion (50–100 millon in average) is not enough for the needs of cellular therapies that would require several billion cells from each cell line for multiple dosing regimens. Amniotic cells proliferate slowly in culture and proliferation rates are significantly higher than rates of cells undergoing apoptosis in the same culture [39]. In this way, Fatimah *et al* have reported that epidermal growth factor (EGF) added to hAECs in culture is able to induce their proliferation and to augment the proportion of cells at S and G2/M phases [40]. They demonstrated that EGF seems to be necessary -but not enough-, in stimulating the growth of cultured hAECs for its application in tissue engineering. Other groups have studied the proliferation of amniotic cells under the treatment with different culture media, reporting that selection of a suitable growth medium is a critical step influencing growth rate of hAECs [41]. In coincidence, other work reported that proliferation capacity of hAECs is sustained by EGF treatment and, without EGF, proliferation goes down to background level [42]. Despite the efforts devoted to studying cell differentiation, many questions concerning the molecular mechanisms of this process still remain to be answered. How hepatic differentiation media regulate the hAECs proliferation and cell cycle progression, expression on pluripotent genes, signaling pathways, apoptosis and senescence, are unknowns to be unravel.

The goal of our work was to study the proliferation and survival of the hAECs during their hepatic differentiation *in vitro*. We have also aimed to determine the change in pluripotency genes and the raise of hepatic markers during the studied process. The precise identification of the mechanisms that govern hAECs proliferation and differentiation into mature hepatocytes could improve the methods to facilitate their application in clinical practice.

## Materials and methods

### Ethics statement

Written informed consent was obtained from all subjects and all study procedures were approved by ethical review committees at the Alejandro Posadas National Hospital (Bioethics Comitte “Dr. Vicente Federico del Giudice”) and the Virgen Macarena University Hospital.

### Amniotic epithelial cells isolation and culture

Human placentas were obtained after cesarean section following normal term pregnancies (37–40 weeks gestation) and immediately suspended in ice-cold PBS and transported to the laboratory. The amnion membrane was manually stripped from the chorion membrane, cut and placed in sterile physiological solution. The amnion was washed two or three times to completely remove bloody or torn pieces and cut into equal 4 pieces. All pieces were sterilized in a laminar flow through successive washings in PBS containing 100 U/ml penicillin and 100 μg/ml streptomycin. Pieces from amnion were digested at 37°C with 50 ml trypsin-EDTA 0.25% to release epithelial cells, during two successive incubations of 20 min. Then, the amnion membrane pieces were removed and the remaining cell solutions were centrifuged 10 min at 1300 rpm. The cell pellet was resuspended and filtered through a 100 μm cell strainer (BD Falcon). Finally, the cell solution was centrifuged (10 min, 1300 rpm) and gently resuspended in IMDM 10% FBS. Cells were stained with trypan blue and counted in a Neubauer chamber. Cell viability and quantity were determined. Sterility of the cultures was determined by seeding 10 μl of cells in a LB plate and incubating them at 37°C. Cells were frozen in 90% FBS or plated for experiments.

Control undifferentiated hAECs were grown in IMDM medium containing 10% FBS and supplemented with 4 mM glutamine, 1 mM sodium pyruvate, 50 U/ml penicillin, 50 μg/ml streptomycin and 1% non-essential amino acids (Invitrogen), at 37°C in 5% CO_2_. Medium was changed twice per week without trypsin treatment (Passage 0).

Control HepG2 cells were grown in DMEM-F12 medium containing 10% FBS, 100 U/ml penicillin, 100 μg/ml streptomycin, 2 mM glutamine, and 1 mM sodium pyruvate, at 37°C in 5% CO_2_.

### Flow cytometry analysis

For evaluation of cell phenotype, cell suspensions were incubated for 20 minutes at 4°C with fluorescein isothiocyanate (FITC) or phycoerythrin (Phy) conjugated antibodies specific for human CD166, CD90, CD326, CD13, SSEA-4, CD45 and Gly-A, or isotype control IgG1. All monoclonal antibodies were obtained from BD Biosciences. Samples were analyzed with a FACSCalibur instrument and the CellQuest software (BD Biosciences).

### Hepatic differentiation of hAECs *in vitro*

Cells were typically cultured for 4–5 days before hepatic differentiation was carried out. To induce the hepatic differentiation we used a two step protocol (modified from [23]). Cells were first initiated for 7 days with IMDM medium 10% FBS, supplemented with 1 mM non-essential amino acids, 1 mM piruvate, 4 mM L-glutamine (Glu), and 10 ng/ml EGF, renewing factor every 3 days in fresh medium. During the next days of the process (7–30), 10 ng/ml EGF and 0.1 μM dexamethasone were added. Differentiation medium was changed every 3 days.

In experiments to determine the ERK 1/2 signaling involvement in proliferation and hepatic differentiation, the MAPKK (MEK) inhibitor PD98059 (10 μM) (Sigma Chemical Company, St. Louis, MO) was added to the corresponding wells 30 min before HD treatment.

### Quantitative real-time PCR assay (qRT-PCR)

Total RNA was extracted from control and treated hAECs using TRISURE reagent, according to the manufacture instructions (Bioline Co). Concentration and purity of the isolated RNA were estimated spectrophotometrically at 260 and 280 nm. For cDNA synthesis, 5 μg of total RNA was reverse transcribed at 50°C during 1 h using the Transcriptor first Strand cDNA synthesis Kit (Roche). *q*RT-PCR reaction was performed using the primers forward and reverse specific for NANOG (F:5’-ATGCCTCACACGGAGACTGT-3’, R:5’-AAGTGGGTTGTTTGCCTTTG-3’), OCT-4 **(**F:5’-GGTGGAGAGCAACTCCAATG-3’, R:5’-TCTGCAGAGCTTTGATGTCC-3’), SOX-2 (F:5’CTCCGGGACATGATCAGC-3’, R: 5’-GGTAGTGCTGGGACATGTGAA-3’), ALBUMIN (F:5’-CCTGTTGCCAAAGCTCGATG-3’, R:5’-GAAATCTCTGGCTCAGGCGA-3’), **α1-**ANTITRYPSIN **(**F:5’-GGAATTCCAGGTTGGAGGGG-3’, R:5’-TGCTCTCCTCAAGCTCTCCT-3’), **α-**FETOPROTEIN (F:5’-CATCCAGGAGAGCCAAGCAT-3’; R:5’-CGCCACAGGCCAATAGTTTG-3’), CYP7A1 (F:5’-TTGCTACTTCTGCGAAGGCA-3’, R:5’-TCCGTGAGGGAATTCAAGGC-3’), CYCLIN D1 (F:5’-AGACCTTCGTTGCCCCTCGT-3’, R:5’-CAGTCCGGGTCACACTTGAT-3’), p21 (F:5’-GATGGCACCAGAGGTGGTTA-3’, R:5’TCCCGAAATATTGGGGAAAG-3’), p53 (F:5’-GGAAGAGAATCTCCGCAAGAA-3’, R:5’-AGCTCTCGGAACATCTCGAAG-3’), CYCLOPHILIN **(**F:5’-CTTCCCCGATACTTCA-3’ R:5’-TCTTGGTGCTACCTC-3’), and GAPDH (F:5’-TCCCTGAGCTGAACGGGAAG-3’, R:5’-GGAGGAGTGGGTGTCGCTGT-3’). Quantitative RT-PCR Master Mix Reagent kit was obtained from Roche (Fast Start universal SYBR Green) and PCR reactions were performed on a Chromo 4 DNA Engine (Bio-Rad). A typical reaction contained 10 μM of forward and reverse primer, 3 μl of cDNA and the final reaction volume was 25 μl. The reaction was initiated by preheating at 50°C for 2 min, followed by heating at 95°C for 10 min. Subsequently, 41 amplification cycles were carried out as follows: denaturation 15 sec at 95°C and 1 min annealing and extension at 60°C. The threshold cycle (CT), from each well was determined by the Opticon Monitor 3 Program. Relative quantification was calculated using the 2^−∆∆CT^ method [43]. For the treated samples, evaluation of 2^−∆∆CT^ indicates the fold change in gene expression, normalized to housekeeping genes (CYCLOPHILIN and GAPDH), and relative to the untreated cells (control). RNA levels in HepG2 cells were considered as positive control for hepatic genes and negative control for pluripotency genes. Melting curves analysis was performed to confirm specificity of amplifications. Reaction mixtures without reverse transcriptase or RNA were run in parallel to ensure the absence of sample contamination.

### Western blot

Cells were incubated in 6-wells plates for the times indicated, with or without differentiation medium. Then, they were washed with 1X PBS. Total cell lysates were prepared in lysis buffer and centrifuged to remove cellular debris. The protein concentration of the supernatant (5μl) was determined by the Bradford staining method [44] with BSA as standard. Lysates were mixed with Laemmli’s sample buffer containing 2% sodium dodecyl sulfate and 30 mM β-mercaptoethanol, boiled for 5 min in cracking buffer, resolved by SDS-PAGE on a 12% gel, and electrophoretically transferred to a nitrocellulose membrane (Hybond; Amersham Pharmacia) thereafter. Membranes were equilibrated in 1X PBS, and nonspecific binding sites were blocked by 5% nonfat milk in PBS at room temperature for 1 h. Then they were immunoblotted with the specific antibody anti-albumin (mouse, 1:1000, Santa Cruz Biotechnology), anti-CYP3A4 (goat, 1:1000, Santa Cruz Biotechnology), anti-CYP7A1 (rabbit, 1:1000, Santa Cruz Biotechnology), anti-Cyclin D1 (mouse, 1:1000, Santa Cruz Biotechnology), anti-p53 (mouse, 1:1000, Santa Cruz Biotechnology), and anti-P-ERK 1/2 (Thr202/Tyr204) (rabbit, 1:1000, Cell Signaling). The antibodies were detected using horseradish peroxidase-linked goat anti-mouse IgG, anti-rabbit IgG or anti-goat IgG (1:1000, Sigma and co.), visualized by the Amersham Pharmacia ECL Chemiluminescence signaling system and a Bio-Imaging Analyzer G-Box Chemi XT4 (Syngene). Control for total ERK 1/2 expression was performed using anti-ERK 1/2 antibody (mouse, 1:1000, Cell Signaling). Control for equal gel loading was carried out by GAPDH detection (mouse, 1:5000, Cell Signaling). Quantification of protein bands was determined by densitometry using Image J ink 1.45 program (National Institute of Health, Bethesda, MD, USA)

### MTT assay

Evaluation of metabolic activity was made with the colorimetric test 3-(4,5-dimethylthia-zolyl-2) 2,5-diphenyltetrazolium bromide (MTT) (Sigma). Metabolically active cells have dehydrogenase enzymes that can cleave tetrazolium ring of MTT and form dark blue formazan crystals that can subsequently be solubilized and quantified by spectrophotometry [45]. At the indicated times, MTT solution (250 μg/ml) was added to all 24-wells plate of an assay and were incubated at 37°C during 30 min. Ethanol 100% was added to all wells and mixed thoroughly to dissolve and extract the dark blue crystals. After a few minutes at room temperature, the plates were read on a microelisa 680x reader (Bio-Rad), at 570nm.

### Immunofluorescence staining

At indicated differentiation times, culture cells were washed with PBS twice and fixed with 4% paraformaldehyde in PBS for 20 min at room temperature. Then, cells were permeabilized with 0.1% Triton-X twice for 10 min, blocked with 2% BSA and incubated overnight with primary antibodies, including anti-SSEA-4 (mouse, 1:100, Cell Signaling), anti-albumin (mouse, 1:100, Santa Cruz Biotechnology), anti-Ki-67 (rabbit, 1:100, Millipore), anti-p21 (rabbit, 1:100, Santa Cruz Biotechnology) and anti-P-ERK (rabbit, 1:100, Cell Signaling). No permeabilization was performed for SSEA-4 detection. Secondary antibodies including FITC-conjugated anti-mouse IgG (goat, 1:100, Sigma) and Alexa Fluor 488-conjugated anti-rabbit IgG (goat, 1:100, Thermo Fisher Scientific) were used according to the manufacturer’s instructions. The samples were incubated at room temperature for 1 h. After further washings with PBS and counterstained with DAPI, samples were mounting with prolong Gold antifading solution (Thermoscientific). In negative controls, primary antibody was omitted for each respective fluorescent tracer (data not shown). Cells were visualized and photomicrographed under an inverted fluorescence microscope (Nikon). Positive FITC or Alexa 488 cells were analyzed and quantified using FIJI-Image J software (Bethesda, MD, USA)

### [H^3^]-thymidine incorporation assay

Amniotic cells were grown in 6-well plates (1 x 10^6^) in complete IMDM medium with 10% FBS or in hepatic differentiation (HD) medium. Immediately after the respective treatment (control or differentiation), cells were incubated with 1 μCi/ml [^3^H]-thymidine (81 Ci/mmol) (Amersham Biosciences) for 18 h. Cells were washed three times with cold water, harvested, and centrifuged for 5 min. The cellular pellet was lysed with 5% trichloroacetic acid (TCA) for 30 min, centrifuged and washed twice with cold PBS. The pellet was resuspended in 150 μl 1M NaOH for 1 h at room temperature. The incorporated radioactivity was quantified by a Beckman scintillation counter (Beckman) and DNA synthesis estimated as dpm/μg protein x h.

### Data analysis

For Western blots analysis, representative images of at least three independent experiments are shown along with the quantification of immunoreactive bands. Quantitative RT-PCR, MTT and [H^3^]-thymidine incorporation assays were repeated separately at least three times to ensure reproducible results. For immunofluorescence analysis, representative images of at least three independent experiments are shown along with quantification of positive fluorescent cells. Results are expressed as the mean ± standard deviation (S.D.). The statistical significance was assessed by ANOVA followed by Bonferroni’s multiple comparisons post hoc test and was calculated using the GraphPad Instat computer program (GraphPad, San Diego, CA). A p value less than 0.05 was considered statistically significant.

## Results

### Amniotic epithelial cells express pluripotency markers that decrease during hepatic differentiation

We have successfully isolated epithelial cells from human amnion, following the described protocol [46] with minor modifications. These cells were isolated with a 95% of purity, determined by flow cytometry (CD166+, CD90-, CD326+, CD13-, SSEA-4+, CD45 +, Gly-A-) (data not shown). First, we observed culture behavior, growth and morphology of cells. *In vitro* hAECs observation under light microscopy (Fig 1A) showed that isolated fresh cells present typical epithelial morphology with rounded shape and high cytoplasm/nuclei proportion in normal maintenance culture. After 3 weeks in normal culture, although they individually maintain their characteristic morphology, they form cellular colonies that increment their size proportionally to time in culture. There is also an increase in cytoplasm size and cell number. In presence of hepatic differentiation (HD) medium, hAECs proliferate robustly from day 3 and on. From day 10 onwards cells become polygonal and granular reaching a confluent monolayer. Amniotic cells morphology begins to be similar to normal human hepatocytes (after 20 days), with some distinguish nucleolus and a few binucleated cells. The size of the differentiated cells was comparable with the size of cultured control hepatic cells (HepG2 cells).

**Fig 1:** HAECs express pluripotency markers and they diminish during hepatic differentiation. **(A)** Amniotic epithelial cells (hAECs) were incubated during 30 days in control medium (C) or treated with hepatic differentiation medium (HD). Representative bright field microscopy images (days 1 and 20) from five independent experiments, at 10X are shown. Scale Bar: 30 μm. **(B)** Isolated hAECs (1 x 10^5^ cells) were plated in complete IMDM medium supplemented with 10% FBS and incubated during 24 h before RNA extraction. RNA from HepG2 cells (Mature cells = MC) was used as negative control expression. **(C)** hAECs were incubated with IMDM 10% FBS (C) or with hepatic differentiation medium (HD) for the indicated times (1,3, 10, 15 and more than 20 days) before RNA extraction. In (**B**) and (**C**), total RNA was extracted as described in Materials and Methods. SOX-2, OCT-4 and NANOG mRNAs were measured by quantitative real time PCR. CYCLOPHILIN and GAPDH were used as internal standards. Results from a representative experiment are shown and expressed as means ± S.D. for five independent experiments performed in duplicates. *p<0.05, **p<0.01 vs. control day 1; ##p<0.01 vs. respective control.

Since hAECs are derived from the pluripotent epiblast, it is reasonable to speculate that these cells might retain pluripotent stem cell characteristics. On this basis, and in order to establish whether hAECs express and maintain the three major pluripotency markers, we measured by *q*RT-PCR, SOX-2, OCT-4 and NANOG genes. Fig 1B shows that hAECs express significant high levels of pluripotency markers, reaching a 370, 42 and 200-fold increase for SOX-2, NANOG and OCT-4 respectively, after 24 hours of culture, compared with mature HepG2 cells. Simultaneously, we performed a two step hepatic differentiation protocol during 30 days and measured the change in stem cell markers expression upon this process. Thus, we examined the expression of the same transcription factors over 30 days in hAECs cultured in control medium (C) or treated with hepatic differentiation (HD) medium. As seen in Fig 1C, OCT-4 and SOX-2 levels significantly increase during the first 10 days in control culture (up to 6 and 12 times respectively) and then begin to diminish. NANOG increments its expression until day 20, reaching a 13,6-fold increase. As expected, in all cases, *in vitro* hepatic differentiation process caused a reduction in pluripotent markers expression, when comparing control with HD in each treatment day (Fig 1C). In control cells, stemness markers are probably influenced by *in vitro* conditions and this may induce their lost in late culture days.

### SSEA-4 expression is down regulated during hepatic differentiation of hAECs

The Stage-Specific Embryonic Antigen-4 (SSEA-4), an early embryonic glycolipid antigen, is an excellent biomarker for the stemness of human cells and is known to be expressed in pluripotent hESCs and in hAECs [9, 47]. In this regard, and in context with previous results (Fig 1), we aimed to measure SSEA-4 expression during normal and HD culture condition. Immunofluorescence analysis (Fig 2) showed that positive expression for SSEA-4 in hAECs was high in normal conditions (80% positive cells) and this expression was retained until day 15 (81% positive cells). Even after long periods of culture (above 20 days) more than 50% of hAECs expressed SSEA-4. However, HD caused a significant decreased in SSEA-4 expression, reaching on average a 30% reduction compared with untreated cells. All these results, confirmed that hAECs possess pluripotency and stemness properties likely downregulated in HD process.

**Fig 2:** Embryonic antigen SSEA-4 diminishes during HD of hAECs. Amniotic cells were seeded in 24-wells plate and incubated in IMDM 10% FBS (C) or hepatic differentiation medium (HD), during indicated times. At each time cells were fixed and SSEA-4 expression (green) was detected using FITC conjugated secondary antibody. Representative micrographs from hAECs at different HD times at 10X are shown. The nuclei were stained with DAPI (blue). Percentage of positive cells is shown on the left of images. Graph on the side shows cells fluorescence intensity for SSEA-4. Scale bar: 30 μm. Representative results from three replicates are shown. ***p<0.001 vs. respective control.

### Specific hepatic markers augment during hAECs differentiation *in vitro*

Since we confirmed that hAECs treated with HD medium lost their stem cell phenotype and acquired a similar hepatic morphology, we aimed to evaluate whether these cells express liver molecular markers. We measured specific hepatic mRNAs expression by *q*RT-PCR. As seen in Fig 3A, HD treatment caused an increase in ALBUMIN, CYP7A1, α-FETOPROTEIN (α-FP) and α1-ANTITRYPSIN (α1-AT) mRNA expression during first 15 days of differentiation, compared with untreated hAECs. Significant expression for all hepatic markers was evident from day 20 and on, with a 20-fold increase for CYP7A1, 8-fold for ALBUMIN, 3544-fold for α1-AT, and 240-fold increase for α-FP (Fig 3B).

**Fig 3:** Hepatic genes expression augments in hAECs with HD treatment. **(A)** Amniotic cells were seeded in 6-wells plate and incubated with complete IMDM medium supplemented with 10% FBS (C) or hepatic differentiation medium (HD) for at least 30 days. At indicated times, mRNA expression of ALBUMIN, α-FETOPROTEIN (α-FP), α1-ANTITRYPSIN (α1-AT) and CYP7A1 was determined. **(B)** hAECs were plated in IMDM 10% FBS (C) or treated with hepatic differentiation medium (HD) and lysated for RNA extraction over 20 days of treatment. In (**A**) and (**B**) total RNA was extracted as described in Material and Methods and hepatic mRNAs were quantified with real time RT-PCR. CYCLOPHILIN and GAPDH were used as internal standards. Representative results from three replicates are shown. *p<0.05, **p<0.01, ***p<0.001 vs. control; #p<0.05, ##p<0.01 vs respective control.

As CYP450 expression is a key marker to determine the presence of hepatocytes like-cells, we measured cytochromes CYP3A4 and CYP7A1 expression by Western blot. CYP3A4 is one of the most important drugs metabolizing enzyme in human liver, whereas CYP7A1 catalyzes the initial step in cholesterol catabolism and bile acid synthesis. They are both markers of definitive endoderm [48, 49]. We also determined albumin expression as a relevant hepatic marker, present not only in fetal but also in adult liver. As seen in Fig 4A, when cells were treated with HD medium, albumin expression was significantly upregulated from the third day and continued rising, reaching a maximum of 12-fold induction on late differentiation (≥ 20 days). Control cells showed low levels of albumin expression probably due to primitive hepatic characteristics of epithelial amniotic cells [21]. Likewise, CYP3A4 and CYP7A1 proteins expression was detected from day three of differentiation onwards (Fig 4B and 4C). As seen in Fig 4B, differentiation medium triggered an increase in CYP7A1, with a maximal 9,6-fold increase on advanced days (≥20). Similarly, CYP3A4 expression augmented on hAECs treated with differentiation factors, from day three and beyond, reaching a 8-fold induction during the last days of the process (Fig 4C). As occurred with albumin, control cells revealed low expression of CYP3A4 and CYP7A1 in early differentiation, confirming hepatic primordial characteristics of freshly isolated hAECs.

**Fig 4:** Hepatic proteins expression augments in hAECs with HD treatment. **(A) (B) (C)** Amniotic epithelial cells were plated in completed IMDM medium with 10% FBS (C) or hepatic differentiation medium (HD) and incubated during at least 30 days. The medium was changed every three days. At indicated times, cell extracts were prepared and proteins were separated on SDS-PAGE gels. Albumin **(A)**, CYP7A1 **(B)**, and CYP3A4 **(C)** expression was determined by Western-blot. Molecular weights were estimated using standard protein markers. Loading controls were performed by immunoblotting the same membranes with anti-GAPDH. Bands densitometry is shown in lower panels. Molecular weight (kDa) is indicated at the right of the blot. Representative results from four replicates are shown. **(D)** Amniotic cells were seeded in 24-wells plate and incubated in IMDM medium supplemented with 10% FBS (C) or hepatic differentiation medium (HD), during indicated times. At each time cells were fixed and albumin expression (green) was detected using Alexa-488 conjugated secondary antibody. Representative micrographs from hAECs at different HD times at 10X are shown. The nuclei were stained with DAPI (blue). Graph below shows positive cells (fluorescence intensity) for albumin. Scale bar: 60 μm. Representative results from three replicates are shown. ***p<0.001 vs. respective control. *p<0.05, **p<0.01, ***p<0.001 vs. control; #p<0.05, ##p<0.01 vs respective control.

In addition, in order to validate all these results we have determined the hepatic differentiation rate (% of albumin positive cells) by immunofluorescence. Fig 4D shows that 67,5% of treated cells are positive for albumin marker on day 10 of HD, and this proportion increases to almost 75% after 20 days of HD, remaining stable. The high differentiation rate obtained confirms the efficiency of the HD treatment on hAECs.

Despite some disparities on HD state, taken together these results demonstrated that hAECs derived hepatic like cells express major early and mature hepatocytes markers.

### Amniotic epithelial cells proliferate during hepatic differentiation

The regulation of proliferation, cell cycle and cell death during hAECs hepatic differentiation are processes barely known till today. It would be relevant to determine when might be the optimal time to hepatic like cells to be transplanted to a damaged liver.

In order to measure the proliferation of amniotic cells during differentiation process we performed [H^3^]-thymidine incorporation assay. We initially evaluated hAECs proliferation during the first 72 hours in control culture condition. As seen in Fig 5A, DNA synthesis reaches 2-fold and 3-fold induction, at 48 and 72 hours respectively, returning to initial values at 96 hours of HD. On the other hand, proliferation was enhanced by HD treatment during the first 72 hours in culture (Fig 5B), with a significant 5-fold induction on day 2 and a 7,5-fold induction on day 3, comparing with untreated control cells. As expected, these control cells increased proliferation up to 3 times at 72 hours in culture. When evaluated thymidine incorporation in later days of HD we found a maximal proliferation rate at day 10 of treatment, and then it decreased up to 1,5-fold induction on day 20 and on. Control cells proliferated at a lower rate all over those days (Fig 5C).

**Fig 5:** Hepatic differentiation increases proliferation and viability of amniotic cells. **(A, B, C)** hAECs were cultivated in 6-wells plate with IMDM 10% FBS (C) or with hepatic differentiation medium (HD). 24 h before indicated times, ^3^H-thymidine (1 μCi/ml) was added and cells were cultured. Cell lysates were prepared and ^3^H-thymidine incorporation was determined as described in Materials and Methods. **(D, E)** Amniotic epithelial cells were seeded (5x10^4^) in 24-wells plate in complete IMDM medium supplemented with 10% FBS (C) or in hepatic differentiation medium (HD). Cells viability was determined by MTT test for up to 72 h **(D)** or during 30 days **(E). (F)** Amniotic cells were seeded in 24-wells plate and incubated in IMDM 10% FBS (C) or hepatic differentiation medium (HD), during indicated times. At each time cells were fixed and Ki-67 expression (green) was detected using Alexa-488 conjugated secondary antibody. Representative micrographs from hAECs at different HD times taken at 10X are shown. The nuclei were stained with DAPI (blue). **(G)** Graph shows the percentage of hAECs positive for Ki-67. Scale Bar: 100 μm. Results from a representative experiment are shown and are expressed as means ± S.D. for five independent experiments. *p<0.05; **p<0.01; ***p<0.001 vs. control.

To further characterize HD effect on amniotic cells, viability experiments were carried out by MTT assay. Fig 5D shows that HD treatment produced an increment in cell viability by 4,4-fold during the first 72 hours of growth. On advanced differentiation days, viability in treated cells was enhanced by 3-fold comparing with control (Fig 5E). Untreated hAECs viability reached a maximal of 2-fold induction during all differentiation process.

As Ki-67 protein is present in the cell nucleus where it only binds the perichromosomal layer in actively growing and dividing cells, it is widely used as a marker to assess cell proliferation. Therefore, we decided to analyze Ki-67 expression during HD of hAECs. We performed immunofluorescence experiments to detect nuclear expression of Ki-67 at day 1, 3, 10 and 20 of differentiation. Results are shown in Fig 5F. HD treatment produced a significant induction of Ki-67 expression during all the process. Quantification of fluorescence intensity shows increments in all cases, with a maximal of 3,5-fold induction on days 3 and 10 (Fig 5G). This effect was stable at least until day 30. These results demonstrate that most of the cells are proliferating when differentiation occurs and this effect is higher in the advanced days of the process. HD medium enhance DNA synthesis, viability and proliferative capacity of amniotic cells making them more competitive for a potential future transplant.

### Cell cycle related proteins expression change during hepatic differentiation process

The molecular mechanisms underlying cell proliferation during HD of hAECs remain unknown. As cell cycle is an integral part of cell proliferation, our next objective was to analyze the expression of Cyclin D1, p53 and p21, key proteins involved in cell cycle, during HD treatment. Cyclin D1 is intimately related to cell proliferation and survival and progression through G1 phase is accomplished by the expression of this cyclin mainly [50]. The p21 protein, a cyclin dependent kinase inhibitor, is involved in the regulation of cell cycle as a major controlling factor at the G1 point. P53 is one of the essential components of the cell cycle that regulates G1/S and G2/M transitions. P21 is the major downstream target of p53 [51]. Cyclin D1 expression analyzed by *q*RT-PCR (Fig 6A) showed a significant increase in treated hAECs, from day 1 and continuously, rising up to 40-fold from day 20 and on. On the contrary, when evaluated p53 gene expression (Fig 6B), we observed a significant 5-fold and 8,3-fold reduction on day 10 and over day 20, respectively, comparing with their untreated controls. Also, p21 expression diminished during hepatic differentiation from day 1 and beyond, reaching a 2,2-fold reduction over day 20 (Fig 6C). Similar results were observed when cell cycle proteins levels were determined by Western blot (Fig 6D and 6E). Cyclin D1 expression increased up to 3-fold on day 15 while p53 expression decreased 2,4-fold after 20 days of HD treatment. Immunofluorescence revealed a 2-fold decrease in p21 expression after 20 days with HD medium (Fig 6F).

**Fig 6:** Human AECs change cell cycle proteins expression during hepatic differentiation. Isolated amniotic cells were seeded in 6-wells plate and incubated with complete IMDM medium supplemented with 10% FBS (C) or hepatic differentiation medium (HD) for at least 30 days. At indicated times total RNA was extracted and mRNA expression of CYCLIN D1 **(A)**, p53 **(B)** or p21 **(C)** were quantified by real time RT-PCR. CYCLOPHILIN and GAPDH were used as internal standards. **(D) (E)** At indicated times, cell extracts were prepared and proteins were separated on SDS-PAGE gels. Cyclin D1 and p53 expression were determined by Western-blot. Molecular weights were estimated using standard protein markers. Loading controls were performed by immunoblotting the same membranes with anti-GAPDH. Bands densitometry is shown in lower panels. Molecular weight (kDa) is indicated at the right of the blot. Representative results from three replicates are shown. **(F)** Amniotic cells were seeded in 24-wells plate and incubated in IMDM medium supplemented with 10% FBS (C) or hepatic differentiation medium (HD), during indicated times. At each time cells were fixed and p21 nuclear expression was detected using Alexa-488 conjugated secondary antibody. The nuclei were stained with DAPI. Percentage of positive cells is shown on the graph. Representative results from two replicates are shown. *p<0.05, **p<0.01, ***p<0.001 vs. control; #p<0.05, ##p<0.01, ###p<0.001 vs. respective control.

All together these results suggest that HD promotes cell cycle progression, increasing S phase entry and favoring proliferation during differentiation. This effect would be favored on the late differentiation days, where they might be especially considered for a hepatic like cells transplantation.

### The MAPK pathway is involved in hepatic differentiation of hAECs

The knowledge about signaling pathways activated during hepatic differentiation of amniotic epithelial cells is limited. MAPKs play important roles in cell growth and differentiation processes. The phosphorylation of ERK 1/2 is closely related to cell survival and proliferation. Thus, we aimed to study changes on the ERK 1/2 MAPK pathways on days 1, 3, 10, 15 and beyond 20 of HD. ERK 1/2 phosphorylation was measured by Western blot. As seen in Fig 7A, ERK 1/2 phosphorylation significantly increase in differentiated hAECs, from the first day of HD and on, up to 10,7-fold after 20 days in culture. Similar results were observed when we detected ERK 1/2 phosphorylation by immunofluorescence. Fig 7B and 7C show that phosphorylation of ERK 1/2 significantly increases with HD medium during all the treatment, reaching a maximal of 1,3-fold increase on day 10, compared with control day 1.

**Fig 7:** ERK 1/2 phosphorylation is stimulated during hAECs hepatic differentiation. **(A)** Amniotic cells were incubated during 1, 3, 10 (top), 15 and up to 30 days (bottom) with IMDM medium 10% FBS (C) or hepatic differentiation medium (HD), as indicated. Extracts from cells were prepared as previously described and loaded in a 12% SDS-PAGE. ERK 1/2 phosphorylation was determined by Western-blot. Loading controls were performed by immunoblotting the same membranes with anti-ERK 1/2 and anti-GAPDH. Bands densitometry is shown in lower panels. Molecular weight (kDa) is indicated at the right of the blot. **(B)** Amniotic cells were seeded in 24-wells plate and incubated in IMDM medium supplemented with 10% FBS (C) or hepatic differentiation medium (HD), during indicated times. At each time cells were fixed and ERK 1/2 phosphorylation (green) was detected using Alexa-488 conjugated secondary antibody. Representative micrographs at 10X from hAECs at different HD times are shown. The nuclei were stained with DAPI (blue). **(C)** Graph shows P-ERK fluorescence intensity in hAECs. Scale Bar: 30 μm. Results are expressed as mean ± S.D. for five independent experiments. *p< 0.05, **p< 0.01, ***p< 0.001 vs. control.

Since activation of MAPK signaling pathway is not necessary link to proliferation, we aimed to evaluate whether ERK 1/2 inhibition changes Ki-67 expression in hAECs during HD. As expected, treatment with PD98059 (a pharmacological MEK inhibitor) caused a downregulation in Ki-67 expression from day 10 and on of HD, measured by Western blot (Fig 8A). Moreover, pharmacological inhibition of MAPK pathway seems to inhibit the hepatic differentiation process. Fig 8B shows that hAECs treatment with PD98059 produced a significant decrease in albumin expression during hepatic differentiation.

**Fig 8:** MAPK signaling pathway participates in proliferation and hepatic differentiation of hAECs. **(A)** Amniotic cells were seeded in 24-wells plate and incubated in IMDM medium supplemented with 10% FBS (C) or hepatic differentiation medium (HD), during indicated times. At each time cells were fixed and Ki-67 expression (green) was detected using Alexa-488 conjugated secondary antibody. Representative micrographs from hAECs at different HD times at 10X are shown. The nuclei were stained with DAPI (blue). Percentage of positive cells (fluorescence intensity) for Ki-67 is shown in the upper right graph. Scale bar: 60 μm. Representative results from three replicates are shown. **(B)** Amniotic cells were incubated during 30 days with IMDM medium 10% FBS (C) or hepatic differentiation medium (HD), with or without PD98059, as indicated. Extracts from cells were prepared as previously described and loaded in a 12% SDS-PAGE. Albumin expression was determined by Western-blot. Loading controls were performed by immunoblotting the same membranes with anti-GAPDH. Bands densitometry is shown in lower panels. Molecular weight (kDa) is indicated at the right of the blot. Representative results from three replicates are shown. ***p<0.001 vs. control; ###p<0.001 vs. respective control.

These results indicate that HD activates the MAPK pathway, probably involved in hAECs survival, proliferation and differentiation process. Further experiments will be needed to establish the MAPK pathway mechanisms involved in the hepatic differentiation of hAECs.

## Discussion

Little is known about the biology of amniotic epithelial cells and even less about the molecular process governing their hepatic differentiation. Some authors have turned their efforts to find the most efficient method to reach such differentiation [31, 36, 52, 53]. However, a few have investigated the mechanisms driving this process and how it could be improved. The human placenta and the extraembryonic tissues have been lately on the focus of regenerative medicine because of the useful properties of their cells in this area. Stem cells derived from placenta have a broad plasticity, immunomodulatory properties, non-tumorigenic risks, non-ethical concerns; they are easy to obtain without invasive and costly procedures and many cells can be acquired in each isolation [3, 54–57]. In recent years, particularly attention has been given to stem cells derived from amniotic membrane. Two types of cells with different plasticity and stemness properties can be isolated from the mesenchymal and epithelial layers of amniotic membranes [37]. Both mesenchymal and epithelial amniotic stem cells have been extensively studied as valuable tools for developing novel therapeutic cell-based approaches [58–61]. Human amniotic epithelial cells are particularly attractive for their clinical use as they are considered pluripotent cells [7]. Since the amnion derives from the early epiblast, before gastrulation occurs, it retains similar pluripotent properties of the embryonic cells. Human AECs can give rise to cell types of all three germ layers [5] but they do not form teratomas when they are transplanted, as embryonic or induced pluripotent stem cells. They are non tumorigenic, since they do not express telomerase [7, 39]. In this way, here we have demonstrated that hAECs express significant levels of the main pluripotency markers, SOX-2, OCT-4 and NANOG, after 24 h of culture. Particularly, this expression remained high during the first 15 days in culture and began to decrease from day 20 and on, indicating that they are loosing stemness properties on advanced days. It is important to note that in order to avoid spontaneous commencement of differentiation during culture or perhaps the epithelial to mesenchymal transition [16] we worked with cells at passage 0. Just freshly isolated hAECs express a high proportion of epithelial markers such as cytokeratins, while mesenchymal markers, generally absent, begin to appear with successive passages [6, 62]. It has been reported that at passages 1 and 2 the expression of these pluripotent markers decreases [63], which make these cells less attractive for a differentiation process.

On the contrary, SOX-2, OCT-4 and NANOG were significantly downregulated in hepatic differentiated hAECs from day 10 of treatment and during the next days. It has been previously reported that those transcription factors are essential to maintain pluripotency through a cooperative interaction [64]. Izumi *et al* [65] have found that the expression of SOX-2 and NANOG is higher in the fetal amnion comparing with term amnion while OCT-4 is maintained. Epiblasts express OCT-4 as long as they remain undifferentiated. Here, we observed that the transcription factors levels are high in recently isolated cells until day 15. After this day, although all genes expression begins to fall, OCT-4 levels go down more abruptly indicating that probably cells loose pluripotency. Thus, it is important to induce the differentiation process immediately after cells isolation. The surface antigen SSEA-4 is found on undifferentiated embryonic cells and is used among other markers to identify stem cells [66]. The epitopes of SSEA-4 appear to play an essential role in compaction of the early human embryo and may enhance integrin activity [67]. In this work we showed that SSEA-4 was downregulated upon hepatic differentiation, from day 1 to 20 and on, but its expression in control cells was kept unchanged. Despite some authors have reported the heterogeneity for cell surface profiling in recently isolated hAECs [6, 63], we found that almost all control cells express the embryonic antigen SSEA-4 (80%) at the beginning of culture and this proportion remains until day 15. These results are similar with those obtained for the pluripotency genes, which also remain high in culture up to day 15. SSEA-4 is an excellent biomarker for stem cells and it is downregulated after differentiation in human ES [68]. Likely, hepatic differentiation caused a decreased in SSEA-4 positive cells going from 62% on day 1 to 7% on advanced days (≥20). These results confirmed that our amniotic epithelial cells have preserved embryonic characteristics similar to those found in hES and as expected, they are lost with the differentiation process. Changes in morphology of isolated cells accompanied this process. During first days in culture, hAECs presented typical cobblestone epithelial morphology. Cells were small and with a rounded shape. As time passed, they proliferated and formed a monolayer. They augmented in size and became giant cells with an increased cytoplasm and formed colonies from day 20 and beyond. In presence of HD medium, amniotic cells proliferated vigorously and formed a monolayer from day 7 and on. They lost epithelial morphology and acquired a hepatocytic polygonal one, with cytoplasmic granules and some multinucleated cells. We confirmed these observations at a molecular level, by determining major hepatic markers expression during 30 days of HD treatment. Hengstler *et al*. [28] have analyzed the necessary criteria in order to establish similarities between hepatic like cells and real hepatocytes. They highlighted that there are certain markers whose induction is easier than others. Detecting cytochromes expression is more difficult than albumin expression. They emphasized the importance of detecting the expression of CYP3A4. Another marker, CYP7A1 has been suggested to be specifically expressed in adult liver, but not in yolk sac cells, being a marker of definitive endoderm [49]. The α-fetoprotein represents the major serum protein expressed by the liver during fetal life, whereas high levels of albumin and CYP3A4 activity are found in hepatocytes from the adult liver [69]. After culture amnion cells with the described hepatic differentiation protocol, they expressed high mRNA levels of both adult and fetal hepatocyte markers: α-FETOPROTEIN, CYP7A1, ALBUMIN, and α1-ANTITRYPSIN. Moreover, from day 20 and beyond these levels became visibly higher. Furthermore, proteins expression of CYP7A1, albumin and CYP3A4 was upregulated after HD treatment. We observed some variations in hepatic markers expression at the beginning of culture probably due to primitive hepatic characteristics of recently isolated hAECs [21]. Hepatic markers expression may oscillate during the first days of treatment due to adaptations to culture conditions, however, in all cases, from day 15 onwards they remained specifically and significantly increased in differentiated cells. The differentiation rate obtained after HD treatment (75%) confirmed the successfulness of the process.

Liver cirrhosis and its associated complications are major causes of morbidity and mortality worldwide [70]. Liver failure may lead to massive hepatic destruction due to repeated and chronic damage to this organ. The common characteristic in this disease is the loss or defective hepatic function and the only curative therapy is orthotopic liver transplant. However, since there is a severe shortage of suitable donor organs, transplantation of human fetal and adult hepatocytes has been investigated and evaluated [27, 71–73]. At present, common sources of human functional hepatocytes include fetal livers and adult marginal livers, both of which are not satisfactory owing to their suboptimal hepatocytic function, culture, cryopreservation and ethical concerns [74]. Replacing hepatocytes with hepatocyte-like cells generated from stem cells is an alternative strategy to overcome the shortage of hepatocytes. Naive hAECs display some relevant features of hepatic progenitors and some characteristic expression of mature hepatocyte markers [21, 75], making amniotic cells attractive as stem cells source for hepatocyte-like cells production. Many studies have focused their efforts on the regenerative properties and differentiation potential of human amniotic membrane stem cells [18, 31, 36, 60, 76, 77], yet, information concerning hAECs biology and/or their hepatic differentiation is rare. As large numbers of differentiated cells would be required for effective transplantation, it would be crucial to improve that process. In this way, a recent study [78] has demonstrated that hAECs and hAMSCs display similar growth ability/day, increasing their proliferation rate until day 5 in culture. In general, one important limitation for amniotic cells is the yield obtain per amnion (5x10^7^ cells) and the poor proliferation in culture [79]. Our results showed that hAECs proliferated during the first 3 days in culture, doubling and tripling their rate at 48 and 72 h respectively. Proliferation rate decreased from day 4. We observed similar results for cell viability. It has been demonstrated that even when hAECs are cultured in growth factor supplemented medium (like platelet derived growth factor, fibroblast growth factor or hydrocortisone) they still do not achieve a considerable increase in growth rate [80, 81]. Fatimah *et al* have reported that in the presence of certain EGF doses hAECs displayed higher growth rate than without it [40]. Other studies on epithelial cells such as epidermal keratinocytes or oropharyngeal keratinocytes have shown similar results [82, 83]. Indeed, some authors have added EGF to culture medium in different concentration in order to promote and maintain cell growth [7, 80]. In our case, hepatic differentiation medium containing EGF (10 ng/ml) in addition to dexamethasone and a rich culture medium, promoted a significant increase in proliferation, growth and viability of hAECs from day 3 and until the end of HD treatment. Proliferation during HD was 5-fold and 7-fold times higher than in control cells, after 48 and 72 h in culture respectively. This effect lasted after 20 days of differentiation. When we cultured cells only with EGF, proliferation was lower than with HD medium and no changes related to hepatic characteristics were detected (data not shown). In agreement, the expression of proliferating cell nuclear antigen, Ki-67, significantly increased in control hAECs and this increment was higher during hepatic differentiation, providing evidence that HD treatment promotes growth of amniotic cells. Indeed, Ki-67 expression indicates progression of differentiated cells in cell cycle, since it is known to start being expressed in the G1 phase, and has increased expression during the S phase [84]. These results demonstrated that differentiation applied to hAECs would be useful not only to produce hepatic like cells but also to improve cell number and proliferation capacity. As follows, we have analyzed some regulators of cell cycle at the mRNA level during differentiation induction. We found that CYCLIN D1 expression was slightly upregulated during the first 15 days of HD comparing with undifferentiated cells, while from day 20 onwards, CYCLIN D1 increase became statistically significant with a 40-fold induction. CYCLIN D1 is one of the positive cell cycle regulators, necessary for G1 to S phase transition, and its concentration increases in dividing cells during the G1 phase [85]. This phase is known to be a permissive phase to initiate cell fate. During G1 phase occurs the transcriptional control of ‘decision’ genes, making cells unresponsive to signals outside this phase [86]. This implies that developmental genes are transcriptionally primed in G1 and that this phase represents a ‘window of opportunity’ for differentiation. We found that Cyclin D1 was upregulated during hepatic differentiation of hAECs, accordingly with the increase of proliferation and survival and with the differentiation state itself. One of the essential components of the cell cycle arrest is p53, “the guardian of the genome”, which regulates the G1/S and G2/M transitions of the cell cycle. Regulated expression of wild-type p53 in p53-null human fibroblasts causes growth arrest in both G1 and G2/M [87]. The p21/WAF1 protein, a cyclin dependent kinase inhibitor, plays a key role in regulating cell cycle via G1 phase control, and is a downstream target of p53. Once activated by p53, p21 inhibits cell cycle by arresting and blocking progress to S-phase through the inactivation of cyclin-dependent kinases and inhibition of proliferating cell nuclear antigen (PCNA) [88]. We have found that p53 and p21 expression is down regulated after a week of HD treatment, reaching maximal reduction after 20 days. Increased Cyclin D1 expression in addition to low levels of p53 and p21 would indicate that amniotic cells are prone to proliferate, after receiving differentiation stimulus, enlarging hepatic like cells number. It has been reported [40] that EGF regulates cell cycle progression of cultured hAECs because of its mitogenic effect. This study demonstrated that HD medium promotes hAECs proliferation through the control of cell cycle genes like p53 and p21, leading the major cells proportion to enter at S and G2/M phase. However, studies about the effect of EGF in combination with dexamethasone, and a specific HD protocol over hAECs cell cycle, proliferation and apoptosis are lacking. Similarly, signaling pathways possibly involved in HD of amniotic epithelial cells remain poorly understood. The MAPKs have been reported as the most important proteins involved in mitogenic signals. MAPK family transduction proteins include ERK, p38 kinase, and JNK, among others [89]. Although p38 and ERK have been shown to play important roles in mediating stem cell proliferation and differentiation [90–92], their specific involvement in the differentiation into hepatocytes remains unclear. The Ras-Raf-MEK-ERK pathway phosphorylates a spectrum of substrates and plays an integral role in cell cycle progression and survival [93]. During G1 phase, cells are responsive to extracellular signaling and, in particular, to mitogenic signaling such as the MAPK pathway, which regulates the activity of Cyclin D and/or CDK4/6 [94]. In addition, the PI3K/AKT and MAPK signaling pathways have been shown to be involved in early liver development and hepatic differentiation [95]. Here, our initial results showed that ERK 1/2 are significantly activated from the beginning of differentiation and last until day 20 and beyond. ERK 1/2 phosphorylation was detected in control cells at early culture times and began to decrease from day 10 and on, probably due to a decline in proliferation rate and the absence of external stimulus. Immunofluorescence analysis revealed similar results where a significant increase of P-ERK 1/2 from day 1 to the end of HD treatment demonstrates MAPK signaling pathway activation. This activation could be related not only to cell growth and proliferation but also to mechanisms associated to hepatic differentiation. In fact, we observed that hAECs incubation with HD in combination with a pharmacological MEK inhibitor (PD98059), interfered in the hepatic differentiation of cells, since albumin expression was significantly diminished after 20 days in culture. Moreover, we determined that ERK 1/2 inhibition caused a significant downregulation of Ki-67 expression during hepatic differentiation, demonstrating the probable involvement of MAPK signaling pathway in proliferation of differentiated hAECs.

MAPK signaling in somatic cells is a potent inducer of differentiation and, in this way, links proliferation and developmental progression in somatic cells [96]. Gao *et al* [95] have determined that the inhibition of ERK by ethanol blocked hepatic differentiation of hESC, indicating that the activation of ERK was critical to direct the hepatic progenitors to differentiate towards hepatocytes under certain differentiation condition. In this work, ERK 1/2 inhibition also caused a reduced level of Cyclin D and a moderate cell cycle arrest at G1/S checkpoint. Other study demonstrated that FGF4 and HGF promote the differentiation of bone marrow mesenchymal stem cells into hepatocytes via the MAPK pathway [97]. Several studies have demonstrated the involvement of MAPK pathway in mediating stem cell proliferation and hepatocyte differentiation [98–101]. Indeed, MAPK cascade is a key transduction pathway controlling the hepatocyte morphology, proliferation and survival, and EGF was found to control these morphogenic and mitogenic effects [102]. To our knowledge, this is the first time the activation of MAPK signaling pathway during hepatic differentiation of hAECs is reported. We have demonstrated that the MAPK signaling pathway may be involved not only in the hepatic differentiation but also in the proliferation of hAECs during that process. It remains to elucidate not only the participation of other proteins involved in this pathway but also the activation of other important pathways related to proliferation and differentiation.

In summary, in this work we have clarified some of the mechanisms involved in hepatic differentiation of hAECs. Particularly, we have demonstrated that a simple HD medium upregulates hAECs proliferation rate, promoting the progression in the cell cycle. The HD treatment caused an increase in cell growth and survival, which would improve the quality and capacity of the hepatic like cells facing an eventual transplant.

Our results provide an opportunity to enhance the process of hepatic differentiation of hAECs, and suggest evidence for their potential application in the treatment of liver diseases via cell therapy or tissue engineering. By examining hAECs behaviour, proliferation and survival, we could be able to evaluate their authentic healing potential and bring amniotic stem cells application to liver disease treatment, closer to reality.
